# Oral Squamous Cell Carcinoma: The Role of BIRC6 Serum Level

**DOI:** 10.1155/2022/5425478

**Published:** 2022-08-18

**Authors:** Morteza Banakar, Shima Torabi Ardekani, Razieh Zare, Mahyar Malekzadeh, Hosein Mirhadi, Bijan Khademi, Dinesh Rokaya

**Affiliations:** ^1^Dental Research Center, Dentistry Research Institute, Tehran University of Medical Sciences, Tehran, Iran; ^2^Health Policy Research Center, Institute of Health, Shiraz University of Medical Sciences, Shiraz, Iran; ^3^Department of Oral and Maxillofacial Pathology, School of Dentistry, Shiraz University of Medical Sciences, Shiraz, Iran; ^4^Shiraz Institute for Cancer Research, Shiraz University of Medical Sciences, Shiraz, Iran; ^5^Department of Endodontics, School of Dentistry, Shiraz University of Medical Sciences, Shiraz, Iran; ^6^Department of Otorhinolaryngology, Khalili Hospital-Shiraz Institute for Cancer Research-Shiraz University of Medical Sciences, Shiraz, Iran; ^7^Department of Clinical Dentistry, Walailak University International College of Dentistry, Walailak University, Bangkok 10400, Thailand

## Abstract

**Background:**

Different factors are involved in the incidence, etiology, metastasis, diagnosis, and treatment of oral squamous cell carcinoma, including apoptosis inhibitor proteins. Baculoviral IAP repeat containing protein 6 (BIRC6) is one of the apoptosis inhibitor proteins contributing to cancer cells' survival in many cancer types with diagnostic and treatment importance. This study is aimed at assessing the serum level of BIRC6 in oral squamous cell carcinoma.

**Materials and Methods:**

In this retrospective cross-sectional study, 60 serum samples were collected from 45 male and 15 female patients with a mean age of 61 years as the case group and 28 serum samples of healthy people as a control group. The serum samples were analyzed using a commercial sandwich ELISA kit.

**Results:**

There were no significant differences between BIRC6 serum levels in patients and healthy subjects. Moreover, we did not observe any significant relationships between BIRC6 serum levels and the patients' demographic or clinical characteristics.

**Conclusions:**

There was no significant difference in serum BIRC6 levels in patients with oral squamous cell carcinoma and healthy individuals. Its use in determining the prognosis of squamous cell carcinoma or considering it a determinant marker in this type of cancer may not have a place. More in-depth studies for evaluating BIRC6 serum levels in oral squamous cell carcinoma patients are recommended for better insight into this protein's role in diagnosing, progression, and prognosis of the disease.

## 1. Introduction

Oral cancers are the most common malignancy in Asian countries and consist of more than 50% of all cancers [1]. Oral carcinoma is the sixth most common malignancy in men and 15^th^ in women [2]. Oral squamous cell carcinoma (SCC) is the most common oral cancer, an invasive epithelial neoplasm, with variable degrees of squamous differentiation, with or without keratinization [3]. In a study on the epidemiology of oral cancers in Iran, SCC, with an average prevalence of 70.0%, is the most common cancer among oral cancers [4]. SCC comprised at least 90 percent of oral neoplasms [5]. When studying the ten-year prevalence of oral cancers in Iran, 48% of all cancers were squamous cell carcinoma [6, 7]. There are 30000 new disease cases and 7400 deaths annually in the United States. However, average yearly incidence and mortality were variable among different races, minorities, sex, and age groups [8, 9].

Different factors are involved in the incidence, etiology, metastasis, diagnosis, and treatment of the SCC, including the apoptosis inhibitor proteins [10]. Baculoviral IAP repeat containing protein 6 (BIRC6) is one of the apoptosis inhibitor proteins, which shows its inhibitory function by binding with preapoptosis factors and leading to an apoptosis inhibitory effect [11]; therefore, it contributes to the survival of cancer cells of many cancer types [12]. BIRC6 exerts its inhibitory effects through binding to caspase and leads to cell resistance like other IAPs proteins such as DIABLO [13]. BIRC6 increases cancer invasion to different tissues, disease recurrence, resistance to different treatments such as chemotherapy, and severity [11]. Therefore, this protein has diagnostic and treatment importance.

The role of BIRC6 in many cancer types has been investigated, including the brain, leukemia, osteosarcoma, colon, and lung [14]. According to previous studies, overexpression of BIRC6 is associated with higher cell proliferation, poorer prognosis, and worse clinical findings at the time of cancer diagnosis [15], in which we can point to the investigation of the role of BIRC6 in colorectal cancer [15], hepatocellular cancer [16], non-small-cell lung cancer [11], epithelial ovarian cancer [17], prostate cancer [18], lung tissue cancers [19], esophageal squamous cell carcinoma [20, 21], gastric carcinoma [22], acute leukemia, and acute myeloblastic leukemia [23]. However, the BIRC6 level has not been studied in oral cancers.

This study is aimed at investigating the presence of BIRC6 as a biomarker in oral squamous cell carcinoma. Determining the role of this marker in oral cancers can significantly impact the prognosis, diagnosis, and treatment of oral cancers.

## 2. Materials and Methods

### 2.1. Subjects

This study was approved by the ethics committee of Shiraz University of Medical Science (IR.SUMS.REC.1397.203). In this cross-sectional study, 60 serum samples from those affected by oral SCC, including 45 male and 15 female patients with a mean age of 61 ± 13 years as a case group, and 28 serum samples of healthy individuals, including 20 men and 8 women with a mean age of 61 ± 13 years as a control group were collected. All participants were hospitalized in the ENT units of the Shiraz Khalili hospital. SCC diagnosis was confirmed histopathologically. Participants who suffered from other malignancies by history, inflammatory, or infectious diseases (in the last three years) have been excluded from the study. The control group consisted of healthy volunteers without any history of cancer, inflammatory or infectious diseases on their own, and first-degree family in the last three years. The informed consent form was completed and signed by all the study participants at the beginning of the study.

### 2.2. Sampling

The blood samples were taken by venipuncture method and then centrifuged at 3,000 rpm for 10 min. Then, aliqouted serum samples were stored at -80°C for future analysis. After completing the sample, the BIRC6 concentrations were measured using a Sandwich ELISA kit (MyBioSource: Baculoviral IAP repeat-containing protein 6 (BIRC6), ELISA Kit) according to the manufacturer's protocol. The ELISA kit contains a 96-well microplate, precoated with the anti-BIRC6 monoclonal antibody. In order to perform the ELISA Sandwich assay, the manual of the MyBioSource BIRC6 ELISA (MBS760993) kit was followed.

### 2.3. Statistical Analysis

We excluded 3 of 88 samples (2 cases and one control) from our calculations because the resulting concentration exceeded the kit's detection range (0.156-10 ng/ml). The BIRC6 concentrations of case and control samples were compared using the Mann–Whitney *U* statistic. Furthermore, the Mann–Whitney and Kruskal-Wallis statistics have been used for testing the association between serum BIRC6 concentration and clinical findings. The *p* value of less than 0.05 was statistically considered significant. Moreover, the correlation between age and BIRC6 concentration was evaluated using Spearman's rank correlation.

## 3. Results

In this retrospective study, SCC clinical samples were used. The demographic characteristics and clinical findings of patients who had been studied for BIRC6 serum levels were summarized in Table 1. The average age of the case (*n* = 60) and control (*n* = 28) was about 61 years, in the 35-88 years age range. The sex distribution of male and female participants of both groups was approximately 3 : 1. There were two exclusions in the case group and 1 in the control group due to highly exceeding the kit's detection range.

Findings showed that the mean of BIRC6 serum levels in SCC cases was 0.313 ± 0.438 ng/ml, which was higher than the control group with a 0.207 ± 0.106 ng/ml difference was not statistically significant (*p* = 0.788). BIRC6 serum levels were 0.20 ± 0.16 and 0.31 ± 0.41 ng/ml in men and women, respectively; however, the difference was not statistically significant between the sexes (*p* = 0.172). Moreover, the BIRC6 serum levels were increased by age, but this increase wasn't statistically significant (*r* = 0.183, *p* = 0.094).  Table 2 shows the correlation between BIRC6 serum levels of the participants.

The results of comparing the BIRC6 concentration and clinicopathological findings of the patients were presented in Table 3. There were not any significant relationships between BIRC6 serum levels and clinical characteristics of the stage, tumor size, metastasis, and site of cancer.

## 4. Discussion

Cancer prognosis is determined based on the different clinical characteristics, response to administered treatments, and cellular or serum markers. One of the proteins which have currently been used as a predictor of different cancer prognoses such as acute leukemia [23], ovarian epithelial cell carcinoma [17], prostate cancer [24], and other cancer types was BIRC6. Successful treatment of various cancer types requires controlling the disease severity and metastasis. In addition to common treatment modalities such as surgery, chemotherapy, and radiation, one of the recommended ways to control the cancer severity and metastasis and prevent lymph node involvement is to control the expression of various genes and proteins such as BIRC6.

This study included 85 participants (58 patients and 27 healthy cases) for BIRC6 serum levels. Findings did not show any significant association between BIRC6 levels of SCC patients and healthy subjects (*p* = 0.172). However, previous studies reported a significant association between the BIRC6 level of patients and healthy subjects, including colorectal cancers [15], lung [19], and prostate cancer [24]. A study by Lee et al. on the association between BIRC6 expression rate and clinical symptoms of esophageal squamous cell carcinoma in 80 patients did not show any significant association between BIRC6 expression rate and variables such as age, sex, size, and differentiation of the cancer cells, while the relationships with lymph node involvement, stage, and metastasis were significant [21]. Our finding did not show any significant correlation between BIRC6 level and age, sex, tumor size, and stage, which was consistent with previous studies. However, we did not observe any significant association between BIRC6 serum levels and clinicopathological variables such as metastasis, lymph node involvement, size, and stage.

As noted, the finding did not show any association between BIRC6 serum level and clinical characteristics of oral squamous cell carcinoma, such as lymph node involvement. Although previous studies have shown a significant association between BIRC6 expression and lymph node involvement in lung cancer, lymphoma, thyroid cancer, and esophageal squamous cell carcinoma, the higher the BIRC6 serum level, the more lymph node involved in the disease. Ma and colleagues found a significant association between BIRC6 expression with cancer metastasis and lymph involvement [25]; however, this is not applicable in oral squamous cell carcinoma. According to our findings, no significant association has been found between the BIRC6 level and metastasis or lymph node involvement.

Because there was no significant relationship between BIRC6 protein and clinical characteristics of this cancer type, we can conclude that BIRC6 may not have any significant role in predicting oral squamous cell carcinoma. Therefore, targeting this protein or corresponding gene may not help in the reduction of oral squamous cell carcinoma severity. This can be due to some limitations that any experimental study can suffer. Despite our precision in performing the study and quantitative measurement of the BIRC6 level using an ELISA kit, many factors such as metabolism, elimination of BIRC6 from blood and serum, and its half-life can impact our results. Moreover, the main purpose of this project was to measure the BIRC6 in blood samples as a low-aggressive low-risk method. Therefore, we recommend a more extensive investigation on BIRC6 expression in the tissue and serum with a bigger sample size of oral squamous cell carcinoma and different test types.

## 5. Conclusion

It showed that the BIRC6 serum level did not have any significant association with age, sex, tumor size, differentiation, metastasis, lymph node involvement, and site of cancer. Moreover, we did not find any differences between patients and healthy subjects regarding BIRC6 serum levels. Therefore, for better generalization, we recommend a more in-depth study of the subject matter using a larger sample size using different molecular tests in order to understand the role of BIRC6 serum level and expression in oral squamous cell carcinoma.

## Figures and Tables

**Table 1:** Frequency distribution of demographic and clinical characteristics of the study participants.

Age	Case (patients)	Mean ± SD	61.32 ± 13.282
		Range	35-88
	Control (healthy)	Mean ± SD	61.14 ± 38.13
		Range	39-86

Sex	Case (patients)	Male/female	45 (75%)/15 (25%)
	Control (healthy)	Male/female	20 (71.4%)/8 (28.6%)

Tumor size	T1/T2/T3	13 (22.4%)/29 (50%)/16 (27.6%)	

Lymph node involvement	0/1/2/3/4	45 (78.9%)/6 (10.5%)/2 (3.5%)/3 (5.3%)/1 (1.8%)	

*N*	N0/N1/N2/N3	45 (77.6%)/5 (8.6%)/8 (13.8%)/0 (0.0%)	

Stage	I/II/III/IV	12 (20.7%)/18 (31.0%)/15 (25.9%)/13 (22.4%)	

Site	Tongue/larynx/salivary glands	20 (34.5%)/34 (58.6%)/4 (6.9%)	

Metastasis		6 (10.31%)	

**Table 2:** The correlation between BIRC6 serum levels of case/control group and male/female participants.

BIRC6 serum levels	Case	0.313 ± 0.438 ng/ml	*p* = 0.788
	Control	0.207 ± 0.106 ng/ml	
	Male	0.20 ± 0.16 ng/ml	*p* = 0.172
	Female	0.31 ± 0.41 ng/ml	

**Table 3:** Correlation between BIRC6 Serum levels and clinical characteristics of the patients.

BIRC6 serum levels	Variable	*p* value
	Tumor size	0.529
	*N*	0.904
	Stage	0.418
	Site	0.136
	Metastasis	0.750

## Data Availability

The data used to support the findings of this study are available from the corresponding author upon request.
